The article "A spatially explicit capture–recapture estimator for single‐catch traps" was published in 2015. Journal: Ecol Evol.

# A spatially explicit capture–recapture estimator for single‐catch traps

**DOI:** 10.1002/ece3.1748

**Published:** 2015-10-19

**Authors:** Greg Distiller, David L. Borchers

**Affiliations:** ^1^ Statistics in Ecology, Environment and Conservation (SEEC)Department of Statistical SciencesUniversity of Cape TownPrivate Bag X3Rondebosch7701South Africa; ^2^ School of Mathematics and StatisticsCentre for Research into Ecological and Environmental ModellingUniversity of St AndrewsThe Observatory, Buchanan GardensFifeKY16 9LZUK

**Keywords:** Density estimation, single‐catch trap likelihood, spatially explicit capture–recapture, statistical methods

## Abstract

Single‐catch traps are frequently used in live‐trapping studies of small mammals. Thus far, a likelihood for single‐catch traps has proven elusive and usually the likelihood for multicatch traps is used for spatially explicit capture–recapture (SECR) analyses of such data. Previous work found the multicatch likelihood to provide a robust estimator of average density. We build on a recently developed continuous‐time model for SECR to derive a likelihood for single‐catch traps. We use this to develop an estimator based on observed capture times and compare its performance by simulation to that of the multicatch estimator for various scenarios with nonconstant density surfaces. While the multicatch estimator is found to be a surprisingly robust estimator of average density, its performance deteriorates with high trap saturation and increasing density gradients. Moreover, it is found to be a poor estimator of the height of the detection function. By contrast, the single‐catch estimators of density, distribution, and detection function parameters are found to be unbiased or nearly unbiased in all scenarios considered. This gain comes at the cost of higher variance. If there is no interest in interpreting the detection function parameters themselves, and if density is expected to be fairly constant over the survey region, then the multicatch estimator performs well with single‐catch traps. However if accurate estimation of the detection function is of interest, or if density is expected to vary substantially in space, then there is merit in using the single‐catch estimator when trap saturation is above about 60%. The estimator's performance is improved if care is taken to place traps so as to span the range of variables that affect animal distribution. As a single‐catch likelihood with unknown capture times remains intractable for now, researchers using single‐catch traps should aim to incorporate timing devices with their traps.

## Introduction

Animal density is a crucial parameter in wildlife management and conservation (Buckland et al. 1993; Marques et al. 2013) and there is often interest in understanding how and why density varies in space (Gaston 2003). Spatially explicit capture–recapture (SECR) models provide a tool for investigating this as they incorporate spatial information on where captures are made (Efford et al. 2009; Royle et al. 2009; Gerber et al. 2012; Noss et al. 2012).

The article "A spatially explicit capture–recapture estimator for single‐catch traps" was published in 2015. Journal: Ecol Evol.

A variety of different detectors or traps are used in capture–recapture or SECR studies. The majority of studies of small mammals use single‐catch traps that catch and hold a single animal at a time (Efford et al. 2009; Krebs et al. 2011; Gerber and Parmenter 2015). Multicatch traps also hold an individual animal until it is released but are able to simultaneously hold multiple individuals. Examples include mist nets for birds and pitfall traps for lizards. Proximity detectors are devices that record the presence of an individual without actually holding it, and unlike the previous two detector types allow an individual to be detected at more than one detector during an occasion. Camera traps, acoustic devices, and hair snares are all examples of proximity detectors.

The characteristics of the type of trap determine the specification of the detection process component of the SECR model (Efford et al. 2009). Capture in either a multicatch or single‐catch trap precludes capture in any other trap during that occasion. The competition between traps for individuals leads to a competing risks formulation for multicatch traps, but single‐catch traps have the additional complexity that once they are full, they are effectively unable to catch any other individuals. A suitable capture model for single‐catch traps therefore needs to account for a second kind of competing risk, that of competition among individuals for traps (Efford et al. 2009). The construction of a suitable likelihood for single‐catch traps is considerably more complicated than for multicatch traps, and to date no likelihood function for single‐catch traps currently exists (Efford et al. 2009; Royle et al. 2013). Consequently, the multicatch trap estimator is typically used for the analysis of single‐catch trap data.

Trap saturation can be calculated as the average proportion of traps that are occupied at the end of an occasion. As explained above, the extent to which the multicatch estimator assumption that traps do not fill up after catching an individual is violated depends on the degree of trap saturation. The multicatch estimator is therefore expected to perform well for low levels of trap saturation.

Efford et al. (2009) conducted simulations that explored the performance of the multicatch trap estimator when applied to single‐catch trap data. Three distributions for the activity centers were considered: a homogenous Poisson distribution, a Neyman–Scott distribution (with clustered centers), and an inhomogeneous Poisson distribution with an east–west linear gradient in density. The fitted model assumed constant density and a half‐normal detection function that uses two parameters ($g_{0}$, which determines detection function height, and *σ*, which determines its range).

The article "A spatially explicit capture–recapture estimator for single‐catch traps" was published in 2015. Journal: Ecol Evol.

They reported that in all cases, even at high levels of trap saturation (of around 86%), the multicatch estimator of both the density and *σ* parameters performed well. There was negative bias in the $g_{0}$ parameter that increased with increasing trap saturation. The only scenario that exhibited slight bias in density (of around −5%) was that with a gradient in the density of activity centers and a high degree of trap saturation. The tentative conclusion was that the multicatch estimator may be sufficiently robust to use with single‐catch traps as long as extreme trap saturation is avoided.

Traditionally, data from live‐trapping studies do not contain actual capture times. However, devices that record times when a trap is triggered are available and have been used by Cowan and Forrester (2012) to study the activity patterns of possums. A continuous‐time SECR model for proximity detectors that record exact capture times was developed by Borchers et al. (2014). With slight modifications, it can be used to obtain a single‐catch trap likelihood. This study presents a single‐catch trap likelihood for situations in which capture times are recorded and uses simulation to compare the performance of the associated likelihood‐based estimator with that of the multicatch estimator under various scenarios.

## Materials and Methods

We assume that the actual times of capture in single‐catch traps are available, and model the process generating detections as a competing hazards survival process (Borchers and Efford 2008) in which “death” corresponds to being caught and all individuals become “alive” again after release. Each individual is exposed to trap‐specific hazards that we assume are at any time independent of the individual's capture history up to that time (although the model is easily extended to estimate different hazard levels before and after first capture as per model $M_{b}$).

The likelihood for single‐catch traps needs to account for the consequences of a trap catching and holding an individual. The first consequence is that the trapped individual cannot be caught at any other trap until it is released, that is, the individual's exposure to detection by all other traps is zero for the remaining period of capture (the competing hazards formulation takes care of this). The second consequence is that the trap in which the individual is held cannot catch any other individuals until the time of release, that is, exposure to that trap for all other individuals is zero.

The article "A spatially explicit capture–recapture estimator for single‐catch traps" was published in 2015. Journal: Ecol Evol.

If we were dealing with proximity detectors, it would be straightforward to handle latent times of capture by integrating times out of the likelihood as done by Barker et al. (2014) (although their model is for abundance rather than density and does not include both time and space). However, the fact that single‐catch traps induce a dependence between individuals complicates matters and means that a high‐dimensional integral would need to be solved.

### Notation

There are *n* unique individuals caught over a survey of duration *T* with an array of *K* traps. If release times are the same for all traps, then this leads to a natural definition of occasion (for discrete SECR models), and the survey duration *T* can be divided into *L* occasions.

As is typical for SECR models, it is assumed that the individuals have fixed activity center locations for the duration of the survey period: $x_{i}$ for the *i*th individual, which is a distance $d_{k}\left(x_{i}\right)$ from trap *k*. Detection probability is a decreasing function of $d_{k}\left(x_{i}\right)$. The number of times the *i*th individual is caught at the *k*th detector is denoted by $\omega_{ik}$, and instead of a capture history of length *L*, we have the capture times of the $\omega_{ik}\;\leq \;L$ captures $t_{ik}\;=\;\left(t_{ik1},\;\ldots ,\;t_{ik\omega_{ik}}\right)$ at trap *k*, and $t\;=\;\{t_{ik}\}$ (*i* = 1,…,*n*; *k* = 1,…,*K*) denotes the set of all detection times.

The hazard function (representing the mean capture rate per unit time) for the *i*th individual and the *k*th trap at time *t* is denoted as $h_{k}\left(t,\;x_{i};\;\theta \right)$ and can depend on both space (in terms of the distance from the trap to the activity center $x_{i}$) and time. ***θ*** is an unknown vector of hazard function parameters. In the absence of other traps and other individuals, the “survivor function” for individual *i* at trap *k* over the whole survey (the probability of individual *i* not being caught in the trap by time *T*) is $S_{k}\left(T,\;x_{i};\;\theta \right)\;=\;\exp\left(-\int_{0}^{T}h_{k}\left(u,\;x_{i};\;\theta \right)\;du\right)$. The combined detection hazard over all traps at time *t* is $h_{\cdot }\left(t,\;x_{i};\theta \right)=\sum_{k=1}^{K}h_{k}\left(t,\;x_{i};\;\theta \right)$, and the overall probability of detection in (0, *T*) over all detectors is $p_{\cdot }\left(x_{i};\;\theta \right)\;=\;1-S_{\cdot }\left(T,\;x_{i};\;\theta \right)$, where $S_{\cdot }\left(T,\;x_{i};\;\theta \right)=\exp\left(-\int_{0}^{T}h_{\cdot }\left(u,\;x_{i};\;\theta \right)\;du\right)$ is the overall survivor function.

The article "A spatially explicit capture–recapture estimator for single‐catch traps" was published in 2015. Journal: Ecol Evol.

In addition to ***θ***,***ϕ*** is the vector of parameters of the Nonhomogeneous Poisson Process (NHPP) governing animal density and *D*(***x***; ***ϕ***) indicates that the density at a point in space depends on both the ***ϕ*** parameters and the spatial coordinate ***x***. For example, if density foll‐ows an exponential east–west gradient then $D\left(x;\phi \right)=\exp^{\beta_{0}\;+\;\beta_{1}\times \;x\;\mathrm{coordinate}}$ and $\phi \;=\;(\beta_{0},\;\beta_{1})$.

### A continuous‐time likelihood for single‐catch traps

The likelihood for ***ϕ*** and ***θ*** is the joint distribution of the number of individuals captured *n*, and the density of the outcomes “$\omega_{ik}$ events, at times $t_{ik1}\;<\;\ldots \;<\;t_{ik\omega_{ikr}}$”, for all *i* and *k*. With single‐catch traps, the survival function term needs to take account of traps having been taken out of action by catching other individuals. Exposure to any particular trap falls to zero as soon as that trap catches any individual, and once an individual is caught in a particular trap, it cannot be caught in any other trap until it is released.

To construct a likelihood with these features, we define an indicator variable $a_{k}\left(t\right)$ that is 1 if trap *k* is unoccupied at time *t* and zero otherwise (*k* = 1,…, *K*), and we define another indicator variable $v_{i}\left(t\right)$ to be 1 if individual *i* is not in a trap at time *t*, and zero otherwise (*i* = 1,…, *n*). (These variables are readily calculated from the observed capture and release times of individuals at each trap.) The hazard function for individual *i* for trap *k* at time *t* is then conveniently written as $v_{i}\left(t\right)a_{k}\left(t\right)h_{k}\left(t,\;x_{i};\;\theta \right)$. The survivor function for individual *i* to time *t* is defined to be $S_{\cdot }\left(t,x_{i};\theta \right)\;=\;\exp\left(-\int_{0}^{t}v_{i}\left(u\right)\sum_{k\;=\;1}^{K}a_{k}\left(u\right)h_{k}\left(u,\;x_{i};\;\theta \right)\;du\right)$.

The likelihood for ***ϕ*** and ***θ*** for single‐catch SECR surveys then becomes:

(1) $$\begin{array}{cc} L(\phi ,\theta |n,t)= & \frac{e^{-\lambda (\phi ,\theta )}}{n!}\prod_{i=1}^{n}\int_{A}D\left(x_{i};\phi \right)S_{\cdot }\left(T,x_{i};\theta \right)\\ & \times \prod_{k=1}^{K}\prod_{r=1}^{\omega_{ik}}h_{k}\left(t_{ikr},x_{i};\theta \right)\;dx \end{array}$$

where $\lambda \left(\phi ,\;\theta \right)\;=\;\int_{A}D\left(x;\phi \right)p_{\cdot }\left(x;\;\theta \right)\;dx$, and the integral is over all possible activity center locations that could have led to a detection on the survey. The term $p_{\cdot }\left(x;\;\theta \right)$ is the overall probability of being caught during the survey, which depends on the combined detection hazard $h_{\cdot }\left(t,\;x;\;\theta \right)$ over the duration of the survey. This in turn depends on $a_{k}\left(t\right)$ (*k* = 1, …, *K*), which depend on random variables (the times of capture in each trap). Calculating $p_{\cdot }\left(x;\theta \right)$ requires taking expectation over these *K* random variables – something that is prohibitively computationally expensive.

The article "A spatially explicit capture–recapture estimator for single‐catch traps" was published in 2015. Journal: Ecol Evol.

Our estimator therefore involves maximizing the above likelihood equation with *λ*(***ϕ***, ***θ***) replaced by $\hat{\lambda }\left(\phi ,\;\theta \right)-.6pt=-.6pt\int_{A}D\left(x;\;\phi \right)-.1pt\exp\left(-\int_{0}^{T}\sum_{k\;=\;1}^{K}a_{k}\left(u\right)h_{k}\left(u,x;\;\theta \right)\;du\right)dx$, which depends on the observed $a_{k}\left(t\right)$ (*k* = 1, …, *K*).

Consequently, the proposed estimator may not be an MLE and may not enjoy the asymptotic properties of MLEs. We evaluate the bias of the estimator and the coverage of a confidence interval estimator based on the observed information, by simulation.

### Simulations

As stated in the introduction, Efford et al. (2009) found that the multicatch model estimator exhibited slight bias when there was a gradient in density, although an estimator with a constant density model was used in those cases and hence both the detection and density components of the model were misspecified. The simulations conducted here use the same form of density model in simulating and estimating and contrast the performance of the multicatch estimator with that of the single‐catch estimator for other kinds of nonconstant density surfaces. We consider a range of NHPPs, with either exponential or quadratic rate parameters as a function of distance east. Table 1 and Figure 1 provide details of the scenarios used in the simulations. Note that scenario 3 in the quadratic simulations is similar to scenario 2 but with the maximum density being shifted from the center of the trap array to the right‐hand side of the array area.

**Table 1:** Details of four different exponential and quadratic scenarios used in the simulations. $D_{\mathrm{Max}}$ is the maximum density (at 4*σ* from the trap array for the exponential simulations), $D_{S}$ refers to the density at the start of the trap array (where the x coordinate is equal to zero), $\overset{¯}{D}$ is mean density, “Unique” is the mean number of unique individuals captured, and “Trap %” refers to trap saturation and is the proportion of traps occupied at the end of each occasion. Means have been rounded off

Simulation Type	Scenario #	$D_{\mathrm{Max}}$	$D_{S}$	$\overset{¯}{D}$	Unique	Trap (%)
Exponential	1	6.00	2.00	2.77	65	94
	2	6.00	1.00	1.79	50	80
	3	6.00	0.50	1.20	36	64
	4	2.00	0.67	0.92	32	60
Quadratic	1	3.68	2.48	2.56	66	96
	2	3.71	0.52	1.30	47	81
	3	3.86	0.03	1.33	42	69
	4	1.49	0.74	0.80	32	63

The article "A spatially explicit capture–recapture estimator for single‐catch traps" was published in 2015. Journal: Ecol Evol.

**Figure 1:** Simulated density surfaces for the four scenarios. The vertical dashed red lines indicate the borders of the trap array.

Except where stated otherwise, all simulations are over 5 × 24‐h occasions (i.e., all trapped individuals are released simultaneously after each 24‐h period) with a 5 × 4 array of traps and use a *σ* of 100 m, trap spacings of 100 m, and a $g_{0}$ of 0.2. For all scenarios, single‐catch trap data with observed capture times are simulated and two estimators (namely the discrete time SECR multicatch trap estimator and the single‐catch trap estimator proposed in this study) used to estimate the parameters of interest. In both cases, the estimators use the correct form of NHPP rate parameter (exponential or quadratic). As explained in Borchers et al. (2014), the hazard function can be specified in a way that links it with the discrete time model to allow the same detection function to be fitted when the performance of the two models are compared. The model parameters are estimated using an integration area constructed with a buffer equal to 4 × *σ*, but the estimated density surfaces are evaluated within the convex hull of the trap array with a buffer of width 2 × *σ* added.

The approach used to simulate single‐catch trap detection times is adapted from a method for simulating competing risks data ((Beyersmann et al. 2009). Individuals compete for traps, and hence, the capture of one individual changes the relative hazards of capture elsewhere for all other individuals. For this reason, the simulation cannot generate capture times for each individual in isolation and needs to move forward with time rather than loop over individuals.

The steps of the simulation are summarized below:

1. A population of individuals from the given NHPP is simulated. Function sim.popn from the R package secr (Efford 2013) was used for this step.
2. The total hazard across all traps for each individual is calculated and used to generate a vector of capture times (one for each individual). We assume a constant hazard through time leading to the density of capture times following an exponential distribution.
3. The minimum capture time from this vector is taken and the rest discarded. If this time is greater than the end of the study the simulation ends, if not the time is taken to be the capture time. The time of release is also calculated and is based on the assumption that all traps are checked and reset on a set time each day (08:00 used in these simulations).
4. The particular trap where the capture event took place is then drawn from a multinomial distribution using the relative hazard at each as yet unfilled trap as the appropriate vector of probabilities, where the relative hazard for the *k*th trap is $\left(h_{k}/\sum_{K}h_{k}\right)$ , and the sum is over all unfilled traps at the given capture time.
5. The total hazard from the remaining traps and the revised trap‐specific relative hazards are recalculated. A new vector of capture times is simulated and the minimum of these times added to the last capture time. If this new capture time exceeds the release time from step 3, the time is discarded and step 2 restarted from the release time, if not it becomes the next capture time and this step is repeated.

The article "A spatially explicit capture–recapture estimator for single‐catch traps" was published in 2015. Journal: Ecol Evol.

The statistical computing language R (R Core Team 2013) is used for the analysis and the R package secr (Efford 2013) used to fit the multicatch models. Computations are performed using facilities provided by the University of Cape Town's ICTS High Performance Computing team (http://hpc.uct.ac.za).

### Model evaluation

The performance of the estimators is evaluated in a variety of ways. Firstly, the relative biases of the predicted mean density over the area ($\hat{D}$) and of the detection function parameters (${\hat{g}}_{0}$ and $\hat{\sigma }$) for both exponential and quadratic simulations, and of the density slope parameter (${\hat{D}}_{\mathrm{slope}}$) for the exponential simulations are calculated. The estimated parameters of the quadratic coefficients are not reported as they are correlated and are more difficult to interpret than the slope parameter of the exponential rate parameter. Secondly, two measures of overall model performance that are based on predicted density at each point in space are calculated and reported, namely the root‐mean‐squared prediction error (RMSPE), and the root‐mean‐squared bias (RMSB). These measures of model performance are calculated for two different areas: the “full” area which extends 2*σ* beyond the trap array, and the “reduced” area which is defined as the area encompassed by the convex hull of the trap array.

The RMSPE and RMSB are calculated as follows:

$$\text{RMSPE}\;=\;\sqrt{\frac{1}{R}\sum_{r\;=\;1}^{R}\left({\text{MSPE}}_{r}\right),}$$

where

$${\text{MSPE}}_{r}\;=\;\frac{1}{M}\sum_{m\;=\;1}^{M}{\left({\hat{D}}_{mr}-D_{m}\right)}^{2}\times \text{cell area},$$

$$\text{RMSB}\;=\;\sqrt{\frac{1}{M}\sum_{m\;=\;1}^{M}{\left({\hat{\overset{¯}{D}}}_{m}-D_{m}\right)}^{2}\times \text{cell area}},$$

where ${\hat{\overset{¯}{D}}}_{m}$ is the mean estimated density at the *m*th point in space (*m* = 1,…,*M*) averaged over the *R* simulations.

The article "A spatially explicit capture–recapture estimator for single‐catch traps" was published in 2015. Journal: Ecol Evol.

## Results

With single‐catch traps, there is an upper limit on the total number of captures over the survey, which is equal to the number of traps multiplied by the number of occasions. With 20 traps and 5 occasions, there are a maximum of 100 captures, and consequently, the mean number of captures for these simulations is equal to the mean percentage trap saturation and only the latter is reported.

Figure 2 presents a set of plots from the exponential simulations that show the estimated density surface from each simulation overlaid on the true density surface. It is apparent that at high levels of trap saturation the multicatch estimator has a tendency to flatten out the estimated density surface. Table 2 and Figure 3 show that the multicatch model underestimates the slope parameter and that the extent of underestimation varies with trap saturation. Table 2 also shows that the relative bias in mean density is similar for the two models. Consistent with the results from the simulations performed by Efford et al. (2009), the $g_{0}$ parameter is negatively biased with the multicatch estimator and again depends on trap saturation while estimates of *σ* are unbiased. Figure 4 shows that the single‐catch model has lower bias in all cases except scenario 4, and there is not much difference between the two models in terms of RMSPE particularly when not extrapolating beyond the trap array.

**Figure 2:** Results from the simulations with an exponential density surface. The black line depicts the true density surface, the gray lines the estimated density surface from each simulation, and the dashed black line the average of the simulations. The vertical dashed red lines indicate the borders of the trap array.

**Table 2:** Simulation of bias in density and detection parameters estimated by the SECR multicatch estimator and the proposed single‐catch estimator when data are from single‐catch traps with 5 and 10 occasions and density follows an exponential gradient. Relative % bias is shown for each parameter followed by the standard error in parentheses. RB($\hat{D}$) is the relative bias in mean density over the area, *F* refers to the full area (with 2 × *σ*) and *R* to the area spanned by the convex hull of the trap array. In all cases, 500 replications were run and converged

Scenario	Model	RB(${\hat{D}}_{\mathrm{slope}}$)	RB(${\hat{g}}_{0}$)	RB($\hat{\sigma }$)	RB(${\hat{D}}_{F}$)	RB(${\hat{D}}_{R}$)
		5 occasions				
1	Multicatch	−62.29% (1.22)	−66.84% (0.37)	−0.77% (0.65)	−2.09% (0.96)	0.71% (0.99)
	Single‐catch	2.54% (2.43)	3.18% (1.04)	0.43% (0.65)	4.30% (1.08)	2.98% (1.03)
2	Multicatch	−42.18% (1.11)	−53.79% (0.46)	0.23% (0.63)	−4.59% (0.95)	0.99% (1.02)
	Single‐catch	2.53% (1.76)	1.67% (0.98)	0.64% (0.62)	4.29% (1.11)	2.44% (1.06)
3	Multicatch	−27.56% (1.16)	−40.08% (0.67)	0.56% (0.67)	−6.13% (1.01)	0.84% (1.10)
	Single‐catch	2.66% (1.56)	6.21% (1.12)	0.58% (0.65)	3.74% (1.27)	1.03% (1.14)
4	Multicatch	−21.04% (2.61)	−32.72% (0.72)	−0.58% (0.67)	1.61% (1.14)	1.79% (1.14)
	Single‐catch	4.00% (3.40)	3.96% (1.06)	−0.27% (0.65)	5.39% (1.21)	2.95% (1.14)
		10 occasions				
1	Multicatch	−47.76% (1.24)	−68.23% (0.20)	−0.79% (0.36)	−2.58% (0.57)	−0.28% (0.59)
	Single‐catch	2.00% (2.05)	0.84% (0.57)	0.21% (0.35)	1.92% (0.61)	1.06% (0.60)
2	Multicatch	−32.75% (1.05)	−54.80% (0.27)	−0.19% (0.35)	−4.84% (0.64)	−0.31% (0.70)
	Single‐catch	−0.09% (1.44)	0.86% (0.54)	−0.16% (0.33)	1.83% (0.72)	1.01% (0.71)
3	Multicatch	−20.08% (0.95)	−43.61% (0.36)	0.63% (0.39)	−5.31% (0.76)	0.19% (0.86)
	Single‐catch	2.33% (1.18)	0.54% (0.63)	−0.11% (0.37)	2.73% (0.88)	1.16% (0.88)
4	Multicatch	−11.67% (2.41)	−35.14% (0.43)	0.00% (0.41)	−0.78% (0.80)	−0.88% (0.82)
	Single‐catch	7.27% (2.88)	1.28% (0.65)	0.19% (0.40)	1.78% (0.83)	−0.06% (0.83)

The article "A spatially explicit capture–recapture estimator for single‐catch traps" was published in 2015. Journal: Ecol Evol.

**Figure 3:** The sampling distributions of the estimates for the slope in the density model from the exponential simulations for both the multicatch and single‐catch estimators. The arrows mark the position of the mean values, and the red arrows show the true values of the slope parameters.

**Figure 4:** Measures of model performance based on predicted density from the exponential simulations with 5 (top row) and 10 occasions (bottom row). Results are given for both the full area (top left and bottom left plots) and the area spanning the trap array (top right and bottom right plots). Standard errors are calculated using the Delta method for the root‐mean‐square prediction error (RMSPE) and bootstrapping for the root‐mean‐square bias (RMSB), and error bars are plotted using two standard errors. The *x*‐axis is ordered by trap saturation (94, 80, 64, and 60%).

For the quadratic simulations, Figure 5 presents the estimated density surface plots, Figure 6 the RMSPEs and RMSBs, and Table 3 the relative biases of the detection function parameters and the mean density estimates. The results are similar to those from the exponential simulations although, in addition to $g_{0}$ being negatively biased, estimates of *σ* from the multicatch estimator tend to be slightly positively biased in scenarios 2 and 3 where the gradient in density is steeper than the other two scenarios. The RMSPE for the single‐catch estimator is noticeably higher than that for the multicatch estimator for scenario 1 which has the flattest quadratic bump, and for scenario 3 when the peak in density is shifted to the side of the trap array. Note that while in general the multicatch estimator again performs worse for higher levels of trap saturation, scenario 2 (and scenario 3 over the reduced area) has more bias than scenario 1 despite having lower trap saturation (81% vs. 96%).

The article "A spatially explicit capture–recapture estimator for single‐catch traps" was published in 2015. Journal: Ecol Evol.

**Figure 5:** Results from the simulations with quadratic density surfaces. The black lines depict the true density surface, the gray lines the estimated density surface from each simulation, and the dashed black line the average of the simulations. The vertical dashed red lines indicate the borders of the trap array.

**Figure 6:** Measures of model performance based on predicted density from the quadratic simulations with 5 (top row) and 10 occasions (bottom row). Results are given for both the full area (top left and bottom left plots) and the area spanning the trap array (top right and bottom right plots). Standard errors are calculated using the Delta method for the root‐mean‐square prediction error (RMSPE) and bootstrapping for the root‐mean‐square bias (RMSB), and error bars are plotted using two standard errors. The *x*‐axis is ordered by trap saturation (96, 81, 69, and 63%).

**Table 3:** Simulation of bias in density and detection parameters estimated by the SECR multicatch estimator and the proposed single‐catch estimator when data are from single‐catch traps with 5 and 10 occasions and density follows a quadratic shape. Relative % bias is shown for each parameter followed by the standard error in parentheses. RB($\hat{D}$) is the relative bias in mean density over the area, *F* refers to the full area (with 2×*σ*) and *R* to the area spanned by the trap array. Any replications that did not converge or estimated negative or very large variances for any parameter were excluded, “Reps” reports the number of included replications

Scenario	Model	RB(${\hat{g}}_{0}$)	RB($\hat{\sigma }$)	RB(${\hat{D}}_{F}$)	RB(${\hat{D}}_{R}$)	Reps
		5 occasions				
1	Multicatch	−69.54% (0.33)	1.80% (0.66)	5.50% (0.98)	−10.04% (0.86)	500
	Single‐catch	3.19% (1.01)	1.28% (0.62)	4.95% (0.97)	1.78% (1.10)	500
2	Multicatch	−57.22% (0.47)	6.98% (0.69)	1.59% (0.90)	−16.56% (0.67)	500
	Single‐catch	4.68% (1.05)	−0.77% (0.51)	2.98% (0.86)	0.56% (0.87)	481
3	Multicatch	−59.58% (0.46)	4.62% (0.74)	−5.02% (0.88)	−5.95% (0.95)	486
	Single‐catch	3.68% (1.09)	1.16% (0.68)	4.79% (1.07)	0.00% (1.24)	457
4	Multicatch	−36.06% (0.67)	1.34% (0.64)	2.69% (1.02)	−5.38% (0.97)	500
	Single‐catch	3.56% (1.05)	−0.06% (0.60)	3.18% (1.00)	2.18% (1.12)	497
		10 occasions				
1	Multicatch	−70.41% (0.20)	0.80% (0.37)	3.31% (0.66)	−7.88% (0.61)	500
	Single‐catch	0.72% (0.58)	0.17% (0.35)	2.48% (0.63)	1.11% (0.73)	500
2	Multicatch	−59.20% (0.28)	7.38% (0.37)	−1.09% (0.63)	−14.70% (0.52)	500
	Single‐catch	0.95% (0.53)	0.33% (0.29)	1.25% (0.62)	0.26% (0.65)	500
3	Multicatch	−60.36% (0.29)	3.89% (0.42)	−5.12% (0.63)	−6.85% (0.72)	500
	Single‐catch	2.62% (0.61)	−0.43% (0.36)	1.46% (0.71)	0.24% (0.85)	498
4	Multicatch	−38.01% (0.41)	1.72% (0.37)	0.64% (0.80)	−5.84% (0.80)	500
	Single‐catch	1.38% (0.62)	0.46% (0.35)	1.21% (0.79)	0.41% (0.91)	500

On average, the single‐catch estimator accurately estimates the true density surface although the occasional replicate overestimates the gradient in density. In some cases, a slight discrepancy between the average estimated density from the single‐catch estimator and the true density can be seen at the edges of the density surface where no sampling occurs. It should be noted that the sample sizes produced by these simulations are not large. The simulations are rerun with 10 occasions, and the results in Figures 4 and 6 confirm that both the RMSPE and the slight bias reduces with larger sample sizes.

The article "A spatially explicit capture–recapture estimator for single‐catch traps" was published in 2015. Journal: Ecol Evol.

## Discussion

### Comparing the estimators

When density is constant, the multicatch estimator is unbiased or nearly so even when the $g_{0}$ parameter is badly negatively biased (Efford et al. 2009). The multicatch estimator ignores the fact that occupied traps are out of action until they are reset. The estimator appears to compensate for this by underestimating the $g_{0}$ parameter. As stated by Efford et al. (2009), this compensator mechanism results in a surprisingly robust estimator of density although the incorrect estimation of $g_{0}$ would still have implications if used in movement or space‐use models.

A nonconstant density surface can lead to high trap saturation in areas of high density but not in low‐density areas. The assumption implicit in the multicatch trap model that traps continue to operate after catching an individual can therefore be badly violated in the high‐density areas leading to density being underestimated in those areas. The consequent underestimation of $g_{0}$ also gets applied to the traps in low‐density areas where trap saturation may not be high, resulting in density being overestimated in low‐density areas.

When density follows an east–west exponential gradient, the multicatch estimator therefore overestimates density where density is low in the west and underestimates density where it is high in the east. These two errors tend to cancel each other out and the estimator of mean density is nearly unbiased although it underestimates density in high‐density areas and overestimates it in low‐density areas. A slight negative bias is evident when evaluating density over the full area due to the steep exponential increase in the eastern part of the true density surface.

The article "A spatially explicit capture–recapture estimator for single‐catch traps" was published in 2015. Journal: Ecol Evol.

A similar thing happens with a quadratic bump in density whereby the multicatch estimator underestimates density around its peak and overestimates density at the edges resulting in a reasonably unbiased estimate of mean density over the full area. However, the estimator is negatively biased for mean density if evaluated over the reduced area since then the error from underestimating density dominates the corresponding error from overestimating density at the edges. This bias is worst when the peak in density is centered on the trap array as in scenarios 1 and 2.

As expected, trap saturation affects the extent that the multicatch estimator underestimates $g_{0}$. However, the steepness of the change in density also plays an important part and can lead to overestimation in *σ* and to the deterioration of the robustness of the multicatch estimator. When the gradient is slight (as with scenario 4 in both types of simulations), the multicatch estimator performs well.

The single‐catch estimator is approximately unbiased for the parameters of interest, and the confidence interval estimator has reasonably good coverage for the parameters of interest (see Table 4). It is clear that the single‐catch trap estimator has lower bias than the multicatch estimator for trap saturations above about 60%, and the estimators have similar RMSPEs.

**Table 4:** Coverage of the parameter and derived density estimates from the single‐catch model for both the exponential and quadratic simulations, and for both 5 and 10 occasions. The Delta method was used to calculate the variance in the derived density estimates

# Occasions	Scenario	Exponential					Quadratic			
		${\hat{D}}_{F}$	${\hat{D}}_{R}$	${\hat{D}}_{\mathrm{slope}}$	${\hat{g}}_{0}$	$\hat{\sigma }$	${\hat{D}}_{F}$	${\hat{D}}_{R}$	${\hat{g}}_{0}$	$\hat{\sigma }$
5 Occasions	1	0.94	0.94	0.93	0.96	0.95	0.95	0.96	0.97	0.95
	2	0.95	0.95	0.97	0.97	0.95	0.97	0.97	0.96	0.95
	3	0.94	0.94	0.93	0.96	0.95	0.95	0.96	0.97	0.95
	4	0.94	0.94	0.93	0.96	0.95	0.95	0.96	0.97	0.95
10 Occasions	1	0.94	0.93	0.95	0.95	0.95	0.95	0.93	0.96	0.94
	2	0.96	0.95	0.95	0.97	0.94	0.93	0.92	0.94	0.95
	3	0.94	0.94	0.98	0.96	0.95	0.95	0.95	0.96	0.98
	4	0.95	0.95	0.94	0.97	0.96	0.95	0.94	0.96	0.96

### Implications for trap design

If the multicatch estimator is used in a single‐catch study, a trap design that lays traps out with trap density roughly proportional to expected animal density in space may avoid higher trap saturation in areas of high density.

The article "A spatially explicit capture–recapture estimator for single‐catch traps" was published in 2015. Journal: Ecol Evol.

Because the single‐catch estimator sometimes estimates density with substantial positive bias when extrapolating beyond the range of explanatory variables spanned by the traps (the variable x in our simulations), it is important that traps adequately span the range of any covariate that is included in the density model. Furthermore, the variance in the single‐catch estimator for density seems to increase when one extrapolates in this way. For example, the RMSPE from the single‐catch estimator is worse compared to the multicatch estimator in the 1st and 3rd quadratic scenarios with 5 occasions. Both these scenarios are characterized by a sampling design where the trap array does not sample from regions where density is changing. A clustered trap design that spans the range of such covariates would facilitate interpolation rather than extrapolation and ameliorate the high variance in the single‐catch estimator.

## Conclusion

If the focus of interest is only overall density or if density is reasonably constant, then the multicatch estimator should perform well. However, this performance deteriorates with high trap saturation and increasing density gradients. Furthermore, the multicatch estimator is poor at estimating the height (but not range) of the detection function and the detection function parameters may be of interest in their own right (for example to inform models of animal movement).

By contrast, the single‐catch estimators of density, distribution, and detection function parameters are found to be unbiased or nearly unbiased in all scenarios considered. If accurate estimation of the detection function is of interest, or if density is expected to vary substantially in space, then there is merit in using the single‐catch estimator.

In the absence of a single‐catch trap likelihood that does not require observed capture times, we recommend that where possible researchers who are using single‐catch traps and are interested in modeling variation in density in space incorporate timing devices and use a single‐catch trap estimator when trap saturation is expected to be above about 60%.

## Conflict of Interest

None declared.
